RETRACTED

# Clinical Observation of Ropinirole Hydrochloride in the Treatment of Parkinson's Disease

**DOI:** 10.1155/2022/3989770

**Published:** 2022-03-17

**Authors:** JingZhou Zhang, Xiaoli Gao, Yuan Chen, Qingxin Kong

**Affiliations:** Chongqing Chemical Industry Vocational College, Changshou, 401220 Chongqing, China

## Abstract

Parkinson's disease is a degenerative disease of the nervous system, which is more common in middle-aged and elderly people. Currently, the incidence of PD is increasing. The disease is a degenerative disease, which is irreversible and requires life-long treatment. Ropinirole hydrochloride can also be used for Parkinson's disease. Therefore, this article conducted research on this; the purpose is to further determine whether the drug can be used for Parkinson's disease. The method used in this article is a method of quantitative analysis and experimental testing. This article selects Parkinson's disease patients from the provincial hospital to conduct investigations and group experiments on these people to test the effects of different levels of ropinirole hydrochloride in the treatment of Parkinson's disease. Experimental data showed that when the dose of ropinirole was 1 mg, its peak concentration reached 24.95 and the clearance rate reached 143.42. This shows that, in the early stage of medication, it has certain benefits in disease control.

## 1. Introduction

At present, the main use of drugs to treat Parkinson's disease is to control its symptoms, rather than to cure the disease fundamentally. With the deepening of scientific research, many new methods for the treatment of Parkinson's disease have emerged. Whether from the perspective of sociology or market economy, they are the main social problems that hinder the sustainable development of the economy. The solution of the PD problem has reached a critical moment.

There are many theoretical results in the research on the treatment of Parkinson's disease and the research on ropinirole. Pingping and Min shared the use of dressings and decoctions in the treatment of difficult cases of Parkinson's disease combined with flatulence and constipation and provided new information, diagnosis, and treatment ideas for similar patients in the future [1]. Yaning et al. said that, at present, the strategy of PD is to treat symptomatically through drugs, surgery, and physical methods, but it cannot be cured [2]. Jie et al. proposed a comprehensive evaluation of the efficacy and safety of ropinirole in the treatment of Parkinson's disease [3]. To this end, this article intends to study the efficacy of ropinirole hydrochloride in Parkinson's disease.

This article first studied ropinirole hydrochloride, expounding its concept, basic function, and pharmacological mechanism. Secondly, it described Parkinson's disease in detail, proposed the mechanism of Parkinson's disease, and explained several common treatment methods. Then, the MRI evaluation of the treatment effect of PD patients was analyzed. Finally, through experimental investigation, experimental tests were conducted on patients suffering from Parkinson's, and relevant data were obtained.

RETRACTED

## 2. Research on Ropinirole Hydrochloride Used in the Treatment of Parkinson's Disease

### 2.1. Ropinirole Hydrochloride

Ropinirole hydrochloride tablets are prescriptions. It belongs to white to light yellow flakes. It is a dopamine receptor agonist that can enhance the effect of dopamine and correct the conduction elements of the central nervous system. It can also relieve the patient's symptoms and maintain the patient's autonomy and mobility. It can be taken alone or with medication. In fact, the dosage is 0.25 mg 3 times a day. According to individual differences in patients, following the doctor's advice, improper use and dosage of the drug can cause side effects, as does ropinirole hydrochloride tablets. Patients who overdose ropinirole hydrochloride tablets will experience systemic symptoms such as peripheral edema, fever, flu-like symptoms, enlarged abdomen, and cardiovascular symptoms such as enlarged heart, aneurysm, angina, coma, aphasia, convulsions, hypotension, or symptoms such as ataxia. Ropinirole hydrochloride tablets should not be used casually because the drug can cause side effects. And the patients on it strictly follow the doctor's instructions. Master the method and dosage of medication, minimize the side effects of medication, and control the condition [4, 5].

This is mainly used to treat early idiopathic Parkinson's disease. The active ingredient in ropinirole hydrochloride tablets is ropinirole hydrochloride, a dopamine receptor agonist that can treat Parkinson's disease. Its pharmacodynamic mechanism is shown in Figure 1.

Differential equation of pharmacodynamic model:

(1) $$\begin{array}{c} D\left(1\right)=-L_{\text{x}}*X\left(1\right), \end{array}$$

(2) $$\begin{array}{c} D\left(2\right)=L_{\text{x}}*X\left(1\right)-\text{BJ}*B, \end{array}$$

(3) $$\begin{array}{c} D\left(3\right)=Lg0*\left(B-B_{g}\right), \end{array}$$

(4) $$\begin{array}{c} G=G_{0}+G_{\max}*\frac{B_{g}}{\left({GB}_{50}+B_{g}\right)}. \end{array}$$

Among them, the absorption rate constant is *L*_x_. BJ stands for apparent clearance rate.

Patients should start with a low dose at the initial stage and never exceed the maximum dose. It is best to follow the doctor's instructions. Ropinirole hydrochloride tablets can cause side effects such as systemic manifestations and cardiovascular symptoms.

RETRACTED

Ropinirole hydrochloride and other agonists should start with a small dose and gradually increase the dose until satisfactory results are achieved without side effects. Although the clinical application is simple and easy to use, it is extremely sensitive to patients and subjective factors. The limitation of the end point directly affects the precise adjustment of the drug dose, impairs the efficacy of PD patients, and even leads to drug-related side effects [6, 7].

### 2.2. Parkinson's Disease

Parkinson's disease is prone to extravertebral system symptoms, endangering the lives of patients. Parkinson's disease is a subtype of psychosis accompanied by multiple occurrences, mainly manifested by symptoms such as mental abnormalities and memory loss. Middle-aged and elderly people are susceptible to the disease, and there is currently no clinical treatment. Clinical treatment is mainly based on drug control of disease development. Parkinson's disease is a common disease in the elderly. Once Parkinson's disease occurs, the patient's ability to take care of itself gradually deteriorates, which is one of the most important factors for the patient's disability. The pathological feature of the diseased tissue of patients with Parkinson's disease is that dopaminergic neurons in the brain have Lewy bodies, which are toxic to neuronal cells, and this substance can cause neuronal degeneration and death. The misfolded conformation of the protein damages the cell, causing neuronal cell death. The conformational state of synuclein plays an important role in the occurrence and development of Parkinson's disease. Its misfolding and abnormal decomposition can damage mitochondria, destroy the cytoskeleton, and become the central link in the pathogenesis of Parkinson's disease. Effective treatments to explain the pathogenesis of Parkinson's disease can also be found at the molecular and cellular levels [8, 9].

Oxidative stress is closely related to the formation of free radicals. In metabolism, under normal circumstances, the cell's antioxidant system can scavenge free radicals and protect the integrity of cell membranes. However, under pathological conditions, a large number of oxidative stress substances damage the dopaminergic neurons of PD patients. At the same time, it initiates the apoptosis pathway during the pathogenesis, destroys the biofilm that causes Parkinson's disease, and promotes the development of the disease. Oxidative stress plays a very important role in the pathogenesis of Parkinson's disease. Oxidative stress can also activate other toxins in the body and can play an important role in the progression of the disease in a variety of ways [10, 11].

RETRACTED

Mitochondria are the structures where cells produce ATP. When cells generate energy, various molecules such as free radicals also appear, which determine the normal function of cells. When mitochondrial function is restricted, it cannot perform its normal function, thereby producing neurotoxic substances, causing the onset of Parkinson's disease [12].

The tolerance of Parkinson's disease patients is mainly determined by the cause of the disease. The tolerance of patients with Parkinson's disease is closely related to the clinical efficacy, which is mainly manifested in the decrease of drug sensitivity, the increase of adverse reactions, and the increase of toxic and side effects. The most significant of these is that drugs cause neurasthenia and cerebral edema. For this type of case, not only the efficacy and safety but also the economic benefits must be considered in the treatment process [13, 14]. Therefore, when choosing a drug, it is necessary to fully combine the medication plan, individual differences, and psychological factors to make a judgment on the evaluation of the drug effect and formulate a reasonable and effective prescription and treatment plan to improve the patient's tolerance and the improvement of the quality of life after the drug. Failure to properly deal with adverse reactions, drug-resistant physiotherapy, and improper administration methods will affect the efficacy and the quality of life of patients after medication. It may also cause other complications in patients to occur, thereby reducing the degree of patients' need to receive such drugs, and clinical recurrences are prone to cause drug failure.

Under pathological conditions, the function of apoptosis is abnormal, and the body initiates the apoptosis program in many ways, leading to apoptosis of dopaminergic neurons. Apoptosis is achieved through two signal transduction pathways: cell surface receptors and mitochondrial apoptosis.

The pathogenesis of Parkinson's disease is related to immune inflammation. Excessive immune inflammation will accelerate the progression of the disease. Therefore, Parkinson's disease is closely related to immune abnormalities. As a neurotransmitter, excitatory amino acids are needed to maintain normal physiological activities, but current research shows that the excessive nutritional effects of excitatory amino acids can cause neuronal toxicity and participate in the occurrence of many diseases, such as neurodegenerative diseases.

At present, the clinical use of drugs to control the symptoms of disease patients has a serious impact on patients. In clinical treatment, Parkinson's patients are mostly treated with western medicine. However, with the continuous deepening of modern research, its adverse reactions have also increased. Clinically, the treatment effect is poor. Therefore, it is necessary to observe the efficacy of Parkinson's patients.

RETRACTED

Parkinson's disease affects people's quality of life and brings great pain to patients. Therefore, the selection of effective drugs is of great value for improving the symptoms of patients and improving the quality of life. Treatment methods such as exercise therapy, drug therapy, surgical treatment, psychological counseling, and nursing care are also very important.

Since levodopa preparations become “ineffective” in the late stages of the disease, other adjuvant drugs are used in most cases. For example, MAO-B inhibitors can not only reduce the dosage of levodopa but also reduce the “opening” phenomenon of levodopa, which has a neuroprotective effect. The effect of dopamine receptor agonists is similar to that of levodopa supplements, so as an alternative medicine, it can be used to delay the healing effect of levodopa supplements, and it can also delay the fluctuation of motor symptoms caused by levodopa supplements [15].

Dopamine receptor agonists are the drugs of choice for early treatment of Parkinson's disease. Since ergot-free DR agonists have no cardiovascular side effects, ergot-free DR agonists are the first choice, especially in patients with early Parkinson's disease. Ropinirole hydrochloride is a typical nonergot DR agonist. Foreign clinical data show that whether ropinirole hydrochloride is used alone or in combination with levodopa in the treatment of early-onset Parkinson's disease, it has shown a good effect, not only in reducing the dose of levodopa but also in reducing levodopa. The dosage of Pakistan may be delayed. The development of complications of Parkinson's disease is caused by levodopa.

### 2.3. MRI Evaluation of the Treatment Effect of PD Patients

The unified scorecard for Parkinson's disease mainly focuses on the changes in subjects' behavior, and these changes often lag behind the changes in the pathophysiological structure of the brain. UPDRS has obvious disadvantages in determining the pathophysiological nature of the onset of Parkinson's disease. Discover organic changes in the pathways of the black striatum. Therefore, clinicians and researchers still lack the imaging technology that can intuitively and sensitively detect the microscopic changes of the deep cell nuclei of PD patients and use this method to evaluate the effects of PD treatment. MRI technology has attracted more and more attention from researchers because of its advantages such as high tissue resolution and ability to analyze brain tissue functions. In recent years, more and more reports have reported the use of new MRI techniques to assess the impact of Parkinson's disease. Therefore, the application and value of the new MRI technology in the evaluation of the treatment effect of PD patients in recent years are introduced as follows.

RETRACTED

Among the many MRI techniques, there are many reports on blood oxygen level-dependent imaging, perfusion-weighted imaging, MRI spectral imaging, and weighted imaging based on blood oxygen sensitivity. As an MRI technology that can be used to monitor brain nerve function, BOLD fMRI technology can sensitively monitor changes in nerve activity in any area of the brain. After the treatment, the neurological function of each area of the brain develops in the brain, and the subtle changes in it can be sensitively recorded by this technology. DBS can improve the network connection between the cerebral motor cortex, increase the BOLD fMRI signal in this area, and use microlesion effect (MLE) to treat patients with Parkinson's disease. The motor cortex will increase significantly, but it will also restore the damaged brainstem function, that is, increase the BOLD signal of the brainstem. After treatment, the BOLD fMRI signal will change significantly in certain areas of the PD patient's brain. The degree of change of BOLD fMRI signal is used to quantitatively evaluate the effect of PD treatment and guide the clinical treatment process of MP. Therefore, this technology may be a new way to measure the effect of Parkinson's treatment.

PWI technology is a technology that uses intravascular contrast agent to perform multiple analyses on selected slices and finally obtains various flow parameters of the contrast agent in the region of interest, such as blood flow and blood volume. This imaging technique can combine functional imaging and morphological imaging. Based on a good anatomical structure, the blood flow parameters of the ROI can be realized, the blood perfusion state of the ROI can be quantified, and the blood flow of the ROI can be quantified. It can sensitively detect diseased tissues. However, PWI technology also has some disadvantages. Due to the long analysis time, it is difficult for patients to accept long-term research. The level of analysis is relatively low, which means that less information is obtained. Because the pathological changes in the brain of patients with Parkinson's disease are also degeneration of dopamine neurons, it is not a vascular disease. Only when the neuronal activity in certain areas of the brain is very clear, the blood will flow to the brain. Therefore, some of the nerve treatment methods mentioned above have difficulty to withstand large changes in blood flow conditions. Therefore, the value of PWI in monitoring the effect of PD treatment is limited.

RETRACTED

DTI technology is a new technology derived from diffusion-weighted imaging in recent years. At this time, the main goal of treating Parkinson's disease patients is to inhibit neuronal damage, prevent neuron loss in the brain, and feed neurons. Therefore, DTI technology is very feasible to detect the changes of nerve fibers in the brain of patients with Parkinson's disease after treatment. Because DTI technology also has the advantages of short scan time and many parameters, more studies will use this technology to evaluate the treatment effect of PD patients.

## 3. Observation on the Clinical Efficacy of Ropinirole Hydrochloride in Parkinson's Disease

### 3.1. Research Objects

#### 3.1.1. Selection Criteria

*(1) Inclusion Criteria*. The diagnostic criteria were diagnosed as primary Parkinson's disease; 40-70 years old regardless of gender; and if you are receiving levodopa plus peripheral decarboxylase inhibitors or other drugs for the treatment of Parkinson's disease and the dose has been stable for at least 30 days.

*(2) Exclusion Criteria*. Exclude patients with severe dementia and dysarthria that interfere with emotional expression.

Exclude people with other serious physical illnesses.

Exclude people with a history of mental illness.

Exclude people with a history of stereotactic brain surgery, nontraumatic rhabdomyolysis, seizures, or drug abuse.

Exclude people with concurrent use of antipsychotics, antidepressants, drugs that can cause extrapyramidal reactions, or other drugs tested within 30 days after baseline.

Exclude people who are unable to complete family diary or who have poor compliance record.

*(3) Exclusion Criteria*. During the study period, the subjects that had poor compliance and were unable to adhere to the medication and psychological counseling required for the study were excluded.

Those who have experienced serious adverse events, complications, and specific physiological changes and can no longer be studied were excluded.

The condition is changing, and the people taking the drug need to change.

The clinician believes that there are other conditions that should be stopped.

### 3.2. Random Grouping Method

The subjects who meet the diagnosis and inclusion criteria are selected regardless of gender and are divided into the control group and the experimental group by random, parallel controlled experiment method. When the cases that meet the inclusion criteria enter the study, the control group will be treated with basic western medicine for Parkinson's disease, and the experimental group will be given the basic medicine for Parkinson's disease combined with traditional Chinese medicine and psychological intervention.

RETRACTED

### 3.3. Experimental Design

At the 4th, 8th, 10th, 14th, and 16th weeks after enrollment in the study, each antiparkinsonian drug and side effects were evaluated through follow-up inspections and home visits, as well as during the “switch” phase.

### 3.4. Analysis of Plasma Samples

Plasma samples are processed in accordance with Part 1 “Sample Processing Technology,” and the plasma samples exceeding the upper limit of quantification of the standard curve are diluted with plasma soil value and measured. Use WinNonlin 6.3 software to calculate the pharmacokinetic parameters.

## 4. Analysis of Experimental Test Results

### 4.1. Plasma Pharmacy Results

People with PD were given ropinirole hydrochloride, and their blood concentrations at different times are shown in Table 1. Before the start, the blood concentrations of different levels of ropinirole hydrochloride in the patients were 0.35, 0.34, 0.11, and 0.05. After four hours, the patient's plasma concentrations of different levels of ropinirole hydrochloride became 0.82, 0.22, 0.15, and 0.08.

As shown in Figure 2, we can find that when the time elapses 1 hour, the blood drug concentration is the highest, reaching 5.01, 3.63, 1.52, and 0.32 in order of Parkinson's disease patients taking different levels of ropinirole hydrochloride. As time goes on in the later stage, the blood drug concentration is getting lower and lower.

### 4.2. The Main Pharmacokinetic Parameters of Patients with Different Doses of Ropinirole

The noncompartmental model of WinNonlin 6.3 software analyzes the blood concentration-time data of different doses of ropinirole and calculates the pharmacokinetic parameters, including elimination half-life, peak time, peak concentration, clearance rate (Cl), and average residence time (MRI), specifically shown in Table 2.

As shown in Figure 3, we can see that when the dose of ropinirole is 1.5 mg, its peak concentration reaches 9.54 and the clearance rate reaches 104.69. When the dose of ropinirole was 1 mg, its peak concentration reached 24.95 and the clearance rate reached 143.42. When the dose of ropinirole was 0.5 mg, its peak concentration reached 5.82 and the clearance rate reached 124.45. When the dose of ropinirole was 0.2 mg, its peak concentration reached 1.19 and the clearance rate reached 129.26.

### 4.3. Analysis of the Correlation between Pharmacokinetics and Pharmacodynamics

According to the experimental research in this article, the BP value change rate obtained by PET scan is used as the drug efficacy index. The BP value change rate obtained by PET imaging in each dose group is shown in Table 3.

RETRACTED

As shown in Figure 4, the side effects of ropinirole seen in this experience include agitation, irritability, hypotension, and slower heart rate when the dose is too high. In pharmacokinetic experiments, there are great differences among individuals in Parkinson's disease, and there are great differences in drug concentration in the body, which may be an important factor affecting the occurrence of side effects.

## 5. Conclusion

With the development of drug treatment for Parkinson's disease and the insoluble side effects and abuse of levodopa, the number of alternative drugs on the market has gradually increased. Dopamine agonists are used alone or as levodopa. Due to the excellent therapeutic effects of alternative medicines, their neuroprotective effects have received extensive attention from the medical community. The research in this paper found that ropinirole hydrochloride has a significant curative effect in the treatment of early Parkinson's disease and can effectively slow down the onset of the disease. But it may also cause adverse reactions to patients. Therefore, the treatment for Parkinson's disease needs to be continually studied.

## Figures and Tables

**Figure 1:** Schematic diagram of the pharmacokinetic mechanism of ropinirole.

**Figure 2:** Blood drug concentrations at different times.

**Figure 3:** Major pharmacokinetic parameters for different doses of ropinirole patients.

**Figure 4:** Correlation analysis of pharmacokinetics and pharmacodynamics.

**Table 1:** Blood drug concentrations at different times.

	1.5 mg	1 mg	0.5 mg	0.2 mg
0	0.35	0.34	0.11	0.05
1	5.01	3.63	1.52	0.32
2	2.36	1.39	0.61	0.18
3	1.13	0.56	0.28	0.08
4	0.82	0.22	0.15	0.08

**Table 2:** Major pharmacokinetic parameters for different doses of ropinirole patients.

	1.5 mg	1 mg	0.5 mg	0.2 mg
Elimination half-life	1.39	1.49	1.84	1.97
Peak time	0.5	0.64	0.96	1.02
Peak concentration	9.54	24.95	5.82	1.19
Average residence time	1.72	2.05	2.24	2.35
Clearance rate	104.69	143.42	124.45	129.26

**Table 3:** Correlation analysis of pharmacokinetics and pharmacodynamics.

	Peak concentration	Area under curve
0	0.56	1.79
10	1.08	1.37
20	2.35	3.64
30	2.76	3.97
40	1.65	2.52
60	3.85	6.12

## Data Availability

The data underlying the results presented in the study are available within the manuscript.
